This article has been retracted.

# Nontraumatic Lesions of the Clavicle in a Paediatric Population: Incidence and Management

**DOI:** 10.1155/2014/261952

**Published:** 2014-10-29

**Authors:** N. D. Clement, G. Nicol, D. E. Porter

**Affiliations:** ^1^Department of Orthopaedics and Trauma, Royal Hospital of Sick Children, 9 Sciennes Road, Edinburgh EH9 1LF, UK; ^2^Royal Infirmary of Edinburgh, Little France EH16 4SA, UK

## Abstract

*Background*. The incidence of paediatric nontraumatic clavicle lesions is unknown and there is limited literature regarding the management of such patients. *Methods*. A review of a prospectively complied radiological database held at the study was conducted for a defined 10-year period. The study centre is the only paediatric service available for a defined catchment population. The case notes of all patients with nontraumatic lesions were reviewed, and the mode of presentation, the diagnostic dilemmas, and the management were recorded. *Results*. A total of 2133 clavicle radiographs were performed during the study period, with only five having a nontraumatic history. The overall incidence of paediatric nontraumatic clavicle lesions was 0.38 per 100,000 per year. Three patients were diagnosed with chronic recurrent osteomyelitis, one with chronic bifocal osteomyelitis, and one with Langerhans cell histiocytosis. All patients with osteomyelitis demonstrated a typical natural history of a chronic relapsing remitting infection. Three underwent bone biopsy; however, no organism was identified. *Conclusion*. This study demonstrated that the incidence of nontraumatic clavicle lesions is small, and those patients presenting with osteomyelitis should not routinely undergo a bone biopsy and close observation with the appropriate antibiotic therapy is advised.

## 1. Introduction

Nontraumatic lesions affecting the clavicle in children are relatively rare and the exact incidence is not known. There is also a paucity of knowledge regarding the most appropriate diagnostic test(s) and management strategy of such patients when they present. A nontraumatic painful swelling of the clavicle in a child should prompt immediate attention. The differential diagnoses of a clavicle swelling are numerous and include condensing osteitis [1], acute/chronic osteomyelitis, chronic recurrent multifocal osteomyelitis (CRMO), sclerosing osteitis [2, 3], and hyperostosis. Fortunately the incidence of malignancy of the clavicle has been demonstrated to be extremely low [4].

There is limited literature concerning nontraumatic lesions of the clavicle, which is probably due to their rarity and therefore conducting large scale studies would be challenging. Previous studies that have been carried out have been done in large tertiary centres with ill-defined catchment areas and in adults. This makes it impossible to establish the size of the denominator population from which a given number of cases has emerged. The largest study conducted in a tertiary centre in New York by Smith et al. [5] reviewed the prevalence of clavicle bone tumours over a 50-year period and isolated only 7 cases under 19 years of age. Although the incidence of malignant clavicular lesions is extremely low [4] establishing a diagnosis to allow an informed clinical decision to be made regarding the management of these atypical lesions is vital. In such cases performing a bone biopsy is advised.

In contrast, for patients who present with typical clinical and radiological findings to suggest osteomyelitis it is debatable whether potentially harmful diagnostic investigations, such as a bone biopsy, should be undertaken [4]. In adults expert radiological opinion has suggested that clinical presentation together with serial imaging is sufficient for diagnosis and a biopsy is not required unless atypical clinical features are present [3, 6]. This is in contrast with the literature on condensing osteitis in which many case reports view biopsy as an obligatory undertaking [2, 7–9]. However, on aggregation of the 13 published reports reviewing over 80 patients of varying ages who have had clavicle biopsies taken for suspect osteomyelitis only two of these reports demonstrated a positive biopsy [2, 3, 7–15]. Furthermore, one of these positive cultures followed an initial negative result and may, in fact, have been due to surgical contamination. For these reasons defining the incidence of osteomyelitis is also very difficult [16].

The aim of this study was to determine the incidence of all nontraumatic paediatric clavicle lesions diagnosed for a defined region over a 10-year period and to describe the management of those patients presenting with osteomyelitis.

## 2. Methods

Ethical approval was obtained for this study from the University of Edinburgh.

Patients were identified retrospectively from a radiological database (MISYS Radiology) held at the study centre for a ten-year period (1998 to 2007), with a minimum of 6 years clinical follow up. All clavicle radiographs performed during this time were identified. Patients who were identified to have undergone a single radiograph during the study period and for subsequent 3 years after this period (until 2010) were excluded. The subsequent 3-year period was to ensure a patient that may have had an initial radiograph during the study period was not excluded due to a second radiograph being performed after the study period. Patients that had more than one clavicle radiograph were extracted for further investigation. This makes the assumption that fractures were likely to have only one radiograph where as other lesions of the clavicle, especially nontraumatic lesion, would be more likely to undergo serial radiographic assessment. The radiological reports of the patients with more than one radiograph were then reviewed, which are recorded in the database. All those patients with fractures were excluded from the cohort leaving radiographs of clavicle swellings. Clinical case notes for these patients were then retrieved and the information regarding the presentation, diagnostic dilemmas, final diagnosis, and management issues relating to these patients were recorded.

The study centre is the only hospital receiving paediatric trauma for a predominately urban population of 779,000, of which 132,465 (17%) were aged 14 years old or less during the study period. All patients from the catchment area who were treated at the study centre or received their initial management outside our catchment area but resided within it were included.

## 3. Results and Discussion

### 3.1. Results

There were 2133 radiographs of the clavicle performed during the study period, and 95 patients underwent more than one radiograph. The radiographic reports and patient notes were reviewed for each of these 95 patients. After excluding fractures only five patients had nontraumatic clavicle lesions. Three of the patients were diagnosed as having chronic recurrent osteomyelitis, one had chronic bifocal osteomyelitis, and one was discovered to have preexisting Langerhans cell histiocytosis.

Population statistics for the catchment area of the study centre demonstrates the population at risk is 132,465. Hence, over the 10-year period of this study, this equates to approximately 1.3 million children-years of observation. During this period the overall incidence of nontraumatic clavicle lesions in the paediatric population was 0.38 per 100,000 per year, with the incidence of chronic osteomyelitis being 0.31 per 100,000 per year and the incidence of Langerhans histiocytosis being 0.08 per 100,000 per year.

A more detailed case note review of the four patients with osteomyelitis was then conducted to discover their mode of presentation, the investigations performed, and the management implemented.

*Case 1.* A 12-year-old boy presented with a tender painful erythematous swelling on the left clavicle. He reported that the pain and the swelling commenced following a rugby injury. Following a radiograph of the clavicle his general practitioner diagnosed a sternoclavicular subluxation. On referral to the hospital multiple diagnoses were considered including trapezius spasm and Sprengel's shoulder (observing that a possible size discrepancy between the scapulae appeared to exist). On examination the boy held his shoulder in an elevated position and there was swelling of the left clavicle which was tender. He had a full range of shoulder movement but with some discomfort on full abduction. No lymphadenopathy was present.

The radiological report of the initial radiograph reported features indicative of osteomyelitis consisting of thickening, expansion, sclerosis, irregularity, and periosteal reaction of the medial end of the clavicle with an adjacent soft tissue swelling in keeping with osteomyelitis. The full blood count (FBC) was normal and the C reactive protein (CRP) was in the upper limits of normal (6 mg/L); however the erythrocyte sedimentation rate (ESR) was elevated at 32 mm/hour.

The patient was initially treated with a three-week course of oral flucloxacillin. This appeared to reduce his symptoms. However over the next two years this became chronic and relapsing in nature, in which five periods of reactivation were successfully treated either with flucloxacillin or, as on two occasions, as advised by microbiology, with co-amoxiclav and fusidic acid. During the attacks the visible swelling would increase in size. Two years following initial presentation a magnetic resonance imaging (MRI) scan was conducted to delineate whether a Brodie abscess had developed. No abscess was observed and that confirmed changes consistent with osteomyelitis: expansion of the medial end of the clavicle with sclerotic, but well defined cortical margins and a reduction in the size of the marrow cavity due to thickening of the cortices. Over the following year the lesion's size diminished indicating that some remodelling had occurred and he has now been symptom free for five years. No biopsy was undertaken during the course of this disease.

*Case 2.* An eight-year-old girl presented with a six-month history of a painful erythematous swelling over the medial aspect of her left clavicle. She also complained of intermittent night pain but denied any loss of appetite, weight loss, or night sweats. The initial radiological examination suggested that there was expansion of the medial two-thirds of the clavicle with extensive periosteal reaction.

A bone biopsy was obtained to try and establish the diagnosis, but this was negative on prolonged culture. However this did not alter the treatment which consisted of a 6-week course of oral flucloxacillin, which resulted in a significant improvement in both the pain and the swelling. She experienced a recurrence 15 months later which again settled following a repeat course of antibiotics. She has been symptom free for further two years since her last clinical follow-up where she was discharged.

*Case 3.* A seven-year-old girl presented with a two-week history of a painful erythematous swelling of the right clavicle. No precipitating cause could be identified. On examination the lesion appeared to be in the medial third of the clavicle and measured approximately 4 cm in size. The swelling was confirmed on radiographic assessment, which demonstrated the typical appearance of osteomyelitis (Figure 1). The initial episode responded to oral flucloxacillin and phenylpenicillin with improvements in both pain and swelling. No biopsy was undertaken due to the typical radiological findings and the fact that the child responded well to antibiotic therapy.

The child experienced multiple relapses which settled with antibiotic treatment. During each remission ESR was found to be elevated and ranged from 36 mm/hour to 93 mm/hour. Following repeated episodes of active disease, over a 22-month period, the osteomyelitis spread to the lateral margin of the clavicle. She also developed a secondary focus 20 months following initial presentation in the mental area of the mandible (mental nerve function appeared unaffected). This was initially detected by a dental practitioner who could not find a dental cause. A diagnosis of presumed bifocal chronic osteomyelitis was made (although clavicular swelling was asymptomatic at this time point).

On presentation of the mandibular swelling a biopsy was taken of both the mandible and the clavicle, neither of which identified a causative organism; however both did show histological changes consistent with osteomyelitis. In addition to this antistreptolysin O and anti-DNase B titres were elevated. This chronic remitting infection ran a course of 52 months with persistent minor swelling of the clavicle. The patient has been symptom free for three years now.

*Case 4.* An eight-year-old girl presented with a 2-week history of a swollen painful erythematous swelling of the medial third of her right clavicle (Figure 2). No history of trauma was recalled. On examination she had a full range of motion of the shoulder although elevation of the arm produced pain in the medial aspect of the clavicle. No lymphadenopathy was present.

Initially alternative diagnoses were considered including a fracture haematoma; however radiographic examination was consistent with changes due to osteomyelitis. This was reinforced by MRI findings which reported features in keeping with infection with considerable soft tissue swelling which was diffuse with an expanded medial half of the clavicle with ill-defined cortices. A bone biopsy was performed which revealed chronic reactive changes with no organisms identified on microscopy or prolonged cultures. The patient's blood results displayed an elevated ESR at 48 mm/hour and CRP of 20 mg/L. The patient was treated initially with a 7-day course of flucloxacillin which initially resolved the acute exacerbation.

During the course of her disease she suffered nine recurrences, each settling following either one or two weeks of treatment with flucloxacillin. In this case the osteomyelitis was found to progress laterally to involve the middle third of the clavicle. Once these episodic recurrences ceased there was substantial remodelling of the clavicle 4 years after initial presentation (Figure 3).

### 3.2. Discussion

This study has illustrated a unique case series of five patients presenting to the study centre with nontraumatic clavicle swellings and represents 1.3 million children-years of observation. The overall incidence of nontraumatic clavicle lesions is small and the majority of cases are due to an infective cause. The presented series of patients with osteomyelitis illustrates that a chronic and relapsing period is endured, and when managed with antibiotic treatment eventual remission can be expected with remodelling of the clavicle. Biopsy of the lesions does not aid in the diagnosis of osteomyelitis, being negative on prolonged culture for the presented series, which was made on clinical symptoms and signs.

A novel aspect of this study was that nontraumatic lesions of the clavicle are different to those found in adults in whom a much more diverse range of pathologies are commonly seen (malignancy, chronic recurrent multifocal osteomyelitis, hyperostosis, and sclerosing osteitis). Four children were diagnosed with osteomyelitis and one was diagnosed with Langerhans cell histiocytosis. In each case of osteomyelitis the clavicle lesion was the presenting complaint whereas in the case of Langerhans cell histiocytosis (LCH) the child had multiple lesions and the clavicular swelling was not the initial presenting symptom. A recent case report of a child with LCH demonstrated the clavicle pain to be the isolated cause of presentation but was not associated with fevers, overlying skin changes, or swelling and the CRP was within normal limits [17]. A biopsy in this case was essential, to make the diagnosis, and was indicated due to atypical presentation to that of osteomyelitis.

In all four cases of osteomyelitis each initially presented with pain and swelling of the medial end of the clavicle. Clement et al. [4] have demonstrated that this region of the clavicle has an extremely low incidence of malignancy based on data sourced from national and regional cancer registries across Europe. Three of the patients diagnosed with osteomyelitis underwent a clavicular bone biopsy to confirm the diagnosis. However neither biopsy identified an organism nor did it alter the management of the patients. All of the patients with clavicular osteomyelitis demonstrated a typical natural history with resolution of symptoms with antibiotic treatment.

The typical natural history of osteomyelitis of the clavicle is of a chronic relapsing and remitting infection which usually starts at the medial end of the bone, causing pain, often worse at night with a visible erythematous swelling. As the infection runs its course and the remodelling phase begins the clavicular swelling begins to regress leaving the clavicle with a more normal appearance (Figure 3). The resolution time in the cases in this study tended to vary but appears to be in the region of several years after the index episode.

Greenspan et al. [3] and Harden et al. [6] demonstrated that biopsy of the clavicle in an adult population is an unnecessary procedure in the presence of typical features of osteomyelitis. The findings from this study support their observations but furthermore confirm them for a paediatric population. The authors suggest that a typical clinical presentation and radiographic signs together with raised inflammatory markers are sufficient to make the diagnosis of osteomyelitis and dictate management (Figure 4). Patients with an atypical presentation or failing to have resolution of their symptoms with antibiotic therapy may warrant further radiographic investigation and potentially a bone biopsy.

A recent review of focal clavicular lesions by Suresh and Saifuddin [18], which included 59 patients referred to a tertiary tumour centre, concluded that the clavicle is not a common site for any particular tumour. In total for all ages 85% of medial third of clavicle lesions were nonneoplastic in nature, and for patients aged less than 20 years of age no neoplastic lesion was diagnosed during the study period. In addition they also demonstrated that no organism was identified for the eleven bone biopsies taken in this age group. Their findings support our study, confirming the rarity of malignant tumours of the medial end of clavicle in children and the failure of biopsy to obtain a causative organism. Although malignancy of medial clavicle is rare this should be suspected for an atypical patient presentation and further imaging such as a MRI scan should be obtained, and if doubt remains a diagnostic biopsy may be considered in this group.

## 4. Conclusion

This study suggests that osteomyelitis affecting the paediatric clavicle is a more homogeneous entity than osteomyelitis seen elsewhere in the skeleton and undertaking a bone biopsy in which there is a typical clinical presentation and findings on radiological examination to support the diagnosis is both unnecessary and unhelpful in producing a management plan. The features necessary to confirm osteomyelitis at this site in child are as follows:

1. a clinical picture of acute inflammation (pain, swelling, erythema, and heat);
2. elevated inflammatory markers;
3. radiological features of an infective or inflammatory process (expansion, loss of normal trabecular pattern, lucency and/or sclerosis, and periosteal reaction);
4. rapid improvement in symptoms (1-2 weeks) with appropriate antimicrobial therapy.

## Figures and Tables

**Figure 1:** A radiograph of the right clavicle for a seven-year-old girl, at the time of presentation, with a two-week history of a painful erythematous swelling over the medial aspect of the clavicle. The radiograph demonstrates marked expansion of the clavicle medially with an associated periosteal reaction.

**Figure 2:** The radiograph of a right clavicle for an eight-year-old girl who presented with a 2-week history of a swollen painful erythematous swelling of the medial third of her right clavicle. The radiograph demonstrates expansion of the clavicle medially with an associated periosteal reaction and sclerosis.

**Figure 3:** The radiograph of a right clavicle for the eight-year-old girl presented in Figure 2 four years after her initial presentation, demonstrating remodelling of the clavicle with eradication of the infection.

**Figure 4:** Proposed stragergy for the management of medial clavicle osteomyelitis in children.
